The article "Results on Certain Biopolymers Using M-Polynomial and NM-Polynomial of Topological Indices" was published in 2023. Journal: Comput Math Methods Med.

# Results on Certain Biopolymers Using M-Polynomial and NM-Polynomial of Topological Indices

**DOI:** 10.1155/2023/4668505

**Published:** 2023-05-29

**Authors:** H. Mohammed Yasin, M. Suresh, Girum Aklilu Abebe, Samuel A. Fufa

**Affiliations:** ^1^Department of Mathematics, College of Engineering and Technology, SRM Institute of Science and Technology, Kattankulathur, 603203 Tamil Nadu, India; ^2^Department of Mathematics, Addis Ababa University, 1176, Ethiopia

## Abstract

Topological indices are numerical descriptors that aid in the prediction of chemical molecules' physiochemical properties and biological actions. It is often helpful to forecast numerous physiochemical attributes and biological actions of molecules in chemometrics, bioinformatics, and biomedicine. In this paper, we establish the M-polynomial and NM-polynomial of some very familiar biopolymers, which are xanthan gum, gellan gum, and polyacrylamide. The uses of these biopolymers can increasingly take the place of traditional admixtures for the application of soil stability and enhancement. We recover the important topological degree-based indices. Also, we give diverse graphs of topological indices and their relations with the parameters of structures.

## 1. Introduction

Although graph theory has a wide range of applications, chemistry is the primary field in which it is used. Topological indices (TIs) are important in chemical graph theory since they provide scientists with a wealth of information relating to the construction of chemical compounds. The topological index is an arithmetical characteristic feature that describes the network topology of a molecule's structure and makes numerous predictions about molecular characteristics (see [1, 2]).

In the past 20 years, several topological indices have been discovered and are being engaged for correlation examination in the fields of bioinorganic chemistry, pharmaceutical medicine, toxicity, and theoretical chemistry. Since TI's characteristic features contain a large data set and a high predictive value, they are routinely utilized in the development of new drugs. The precision of the physicochemical attributes for chemical compounds determines the uniqueness of the QSAR/QSPR model. These models depend on a few variables, including the choice of the appropriate molecule, the appropriate descriptor, and the appropriate algorithm or modelling tool (see [3–5]).

After Wiener [6] introduced the Wiener index in 1947, topological indices began to advance. Since then, this study has drawn the attention of other scholars and led to the creation of numerous new topological indices. The numerical descriptors are widely utilized because they illustrate how a compound's physical structure and chemical characteristics relate to one another. In the beginning, Wiener used the topological index on QSPR, representing that it worked well along an alkane's boiling point [6]. It was then used to depict a variety of chemical and physical properties of compounds, as well as to connect their structure to biological functions (refer to [7]).

The generalized Randic index was proposed by Bollobás and Erdös [8]. The Randic index was replaced by the harmonic index, which was established by Fajtlowicz. Gutman and Trinajstić [9] found the first degree-based molecular descriptor in 1972, which was known as the Zagreb index in recent days. In 1975, Randic [10] invented the branching index, which was later renamed as connectivity index which characterizes the molecular branching. In recent days, most of the authors refer it as the Randic index. For the molecules, the total *π*-electron energy can be calculated using these topological indices, which are the oldest ones. It is later reformatted and given the name “second modified Zagreb index” by Miličević et al. [11].

Ranjini et al. [12] defined the redefined Zagreb indices. For estimating the heat of production of alkanes, the most accurate method is the augmented Zagreb index. The graph's forgotten index (F-index) was first presented by Gutman and Trinajstić [9] in 1972. A detailed study was carried out by Gutman and Trinajstić. The performance of the index's forecast is very similar to that of the original Zagreb index. Symmetric division is a specific indication of the collective surface area of octane isomers, which has a standard of simple, peculiar, and amusing structure in the developed extremal graphs. Inverse sum index is a representation of aggregate surface area for polychlorobiphenyls (PCBs) (see [13, 14]).

Different physicochemical qualities can be predicted with excellent accuracy using neighborhood degree sum-based topological indices. The third iteration of the Zagreb index was developed by Ghorbani and Hosseinzadeh using the neighborhood degree of the apexes in a specific network.

Researchers have conducted extensive research on surface compaction, drainage techniques, vibration methods, precompression, consolidation, grouting and injection, chemical stabilization, soil reinforcement, and the use of geotextiles and geomembranes in historic cultures. For storage of water, river flooding management, and meeting other basic demands, ancient civil engineering techniques used binders and natural resources. Roman concrete, a mixture of a natural pozzolan substance, aggregates, and a binder such as lime or gypsum, was widely used to build and study structures in ancient Rome (see [15]). Ringelberg et al. [16] find that during the Post Industrial Revolution, for the stabilization of soil, ordinary Portland cement was designed. Postwar rebuilding led to the development of chemical combinations and industrial results. The environmental discrepancies are being smoothed out with the help of engineering fields after the Kyoto Protocol. The unselective improvement has led to environmental degradation, because of which sustainable technology was established. The excessive usage of regular Portland cement and its independence in use have led to a negative influence on the environment. The cement had a number of benefits for building, and it was completely reliable. One of the biggest issues that arose during the manufacturing of cement was the emission of CO_2_, a primary source of greenhouse gases. This has led to a focus on biomediated soil improvement methods by the geotechnical engineers to control the emission of CO_2_. Potentially environmentally friendly alternatives for soil treatment involve environmentally friendly materials and procedures (see [17]). More studies with experimental data and analysis have recently been published (refer to [18–26]). Additionally, microscopic interparticle interactions have been found to increase the bonds between joint biopolymers and soils.

## 2. M-Polynomial and NM-Polynomial

Polynomials are one of the many graph theory techniques that play an important role in applications; the reader may refer to [27, 28]. Hosoya [29] introduced the Hosoya polynomial, which is important for distance-grounded topological indices. M-polynomial was introduced by Deutsch and Klavžar [30], which is one of the two new tools introduced in recent years. NM-polynomial, introduced by Mondal et al. [31], is critical for starting closed methods of various degree-based topological indices. The polynomial that generates the most useful topological indices is the M-polynomial. Because this research is moving so quickly, new indices are created on a daily basis. Recently, several researchers have focused on neighborhood degree sum-based indices, which has increased interest in and led to considerable research on NM-polynomials. The M-polynomial function for degree-constructed indices is paralleled with the NM-polynomial tool. The TIs are derived from the M-polynomial in its generalized form. Similarly, a comprehensive polynomial is derived from the neighborhood degree-based index concept of the NM-polynomial.

The M-polynomial and NM-polynomial of the structure of the biopolymer are calculated; following this, we deduce the many physical and chemically substantial indices and also the neighborhood of those indices.

In general, the definition is used to generate connection indices. Finding a compact method to generate numerous topological indices from a single polynomial is always preferable. The M-polynomial mentioned above is one such approach. The investigation of the properties of the M-polynomial will give perception in the study of topological indices (degree-based). Around the world, there have been numerous investigations on topological indices employing the M-polynomial and NM-polynomials of the graphene structure (see [32–36]).

In this article, an attempt is made in calculating M-polynomial and NM-polynomial for biopolymer structures followed by deriving most physically and chemically significant indices, viz., first Zagreb index *M*_1_(*G*), second Zagreb index *M*_2_(*G*), modified second Zagreb index *mM*_2_(*G*), third redefined Zagreb index *ReZG*_3_(*G*), forgotten index *F*(*G*), Randic index *R*(*G*), inverse Randic index *RR*(*G*), symmetric division index *SDD*(*G*), inverse sum index *I*(*G*), harmonic index *H*(*G*), and its neighborhood versions of the above indices.

## 3. Preliminaries

We begin with some basic definitions which will be applied in the sequel.

In 2015, Deutsch and Klavžar [30] formulated the notion of M-polynomial as follows:

**Definition 1 .**

Let *R* be the simple connected graph, and the *M*-polynomial is defined as

(1) $$\begin{array}{c} M\left(R;x,y\right)=\underset{p\leq q}{\sum }m_{pq}\left(R\right)x^{p}y^{q}. \end{array}$$

In this, *m*_*pq*_ denotes the number of edges *uv* ∈ *E*(*G*), where *d*_*u*_, *d*_*v*_ = (*p*, *q*), respectively. Here, *d*_*u*_, *d*_*v*_ denotes the degree of the vertices *u* and *v* in the graph, respectively.

Mondal et al. [37] introduced the concept of neighborhood M-polynomials in 2020, which is as follows:

**Definition 2 .**

For a simple connected graph *R*, the *NM*-polynomial is defined as

(2) $$\begin{array}{c} NM\left(R;x,y\right)=\underset{p\leq q}{\sum }\chi_{pq}\left(R\right)x^{p}y^{q}. \end{array}$$

In this, *χ*_*pq*_ denotes the number of edges *uv* ∈ *E*(*G*), where *nd*_*u*_, *nd*_*v*_ = (*p*, *q*), respectively. Here, *nd*_*u*_, *nd*_*v*_ denotes the degree of the vertices *u* and *v* in the graph, respectively.

We tabulate the several degree-based and neighborhood degree-based topological indices for the M-polynomial and NM-polynomial in Table 1.

For the degree-based TIs, *δ*_*u*_ = *d*_*u*_, *δ*_*v*_ = *d*_*v*_, and *M*(*R*; *x*, *y*) = *h*(*x*, *y*), and for the neighborhood degree-based TIs, *δ*_*u*_ = *nd*_*u*_, *δ*_*v*_ = *nd*_*v*_, and *NM*(*R*; *x*, *y*) = *h*(*x*, *y*) (Table 1).

Some neighborhood degree sum-based and degree-based TIs and its collection with neighborhood and M-polynomial for the graph *R* are in Table 1, respectively.

(3) $$\begin{array}{c} D_{x}=x\left(\frac{\delta \left(h\left(x,y\right)\right)}{\delta x}\right),\\ D_{y}=y\left(\frac{\delta \left(h\left(x,y\right)\right)}{\delta y}\right),\\ {\left.J\left(h\left(x,y\right)\right)=\left(h\left(x,y\right)\right)\right|}_{y=x},\\ S_{x}=\int_{0}^{x}\frac{{\left.h\left(x,y\right)\right|}_{x=t}}{t}dt,\\ S_{y}=\int_{0}^{y}\frac{{\left.h\left(x,y\right)\right|}_{y=t}}{t}dt. \end{array}$$

## 4. Methodology

The work deals with neighborhood degree sum-based indices for xanthan gum, gellan gum, and polyacrylamide structures. First of all, the NM-polynomials of the structures are calculated, and then, utilizing some calculus operators, various degree sum-based indices are recovered. We use the combinatorial computation, edge partition method, and graph theoretical tools to obtain the outcomes. The graphical representations of the outcomes and comparative study of the findings are performed via 3D plotting and shown by utilizing the MATLAB software.

## 5. Main Results

In this section, we give our key analytical results and divide the sections into three subsections: Xanthan Gum, Gellan Gum, and Polyacrylamide.

### 5.1. Xanthan Gum

Chang et al. discovered an anionic polysaccharide called xanthan gum produced by the bacterium Xanthomonas campestris. It is extremely viscous and is stirred by both hot and cold water. By blocking soil pores, xanthan gum is used in geotechnical engineering to make sandy soils less permeable while also improving soil erosion resistance, as developed by Gioia and Ciriello [38]. Chang et al. [17] demonstrated that treating Korean red-yellow soil with a modest amount of xanthan gum increased soil erosion resistance and promoted vegetative culture. Now, we see the structure of xanthan gum, which is given Figure 1.

From Figure 1, we partitioned the edge for the degree-based indices as shown in Table 2.

#### 5.1.1. M-Polynomial for the Graph of Xanthan Gum

Let *R*_1_ be a molecular graph for xanthan gum; by applying Table 2 in equation (1), we get

(4) $$\begin{array}{c} 10{nxy}^{2}+\left(27n+1\right){xy}^{3}+4{nxy}^{4}+\left(53n-1\right)x^{2}y^{3}+2{nx}^{2}y^{4}+43{nx}^{3}y^{3}+2{nx}^{3}y^{4}. \end{array}$$

#### 5.1.2. Degree-Based TIs of Xanthan Gum Graph Utilizing M-Polynomial

By using equation (4), we calculated the degree-based topological indices for the xanthan gum graph, and the results are as follows:

(5) $$\begin{array}{c} \left(D_{x}+D_{y}\right)f\left(x,y\right)=30nxy^{2}+4\left(27n+1\right)xy^{3}+20nxy^{4}+5\left(53n-1\right)x^{2}y^{3}+12nx^{2}y^{4}+258nx^{3}y^{3}+14nx^{3}y^{4},\\ \left(D_{x}D_{y}\right)f\left(x,y\right)=20nxy^{2}+3\left(27n+1\right)xy^{3}+16nxy^{4}+6\left(53n-1\right)x^{2}y^{3}+16nx^{2}y^{4}+387nx^{3}y^{3}+24nx^{3}y^{4},\\ \left({D_{x}}^{2}+{D_{y}}^{2}\right)f\left(x,y\right)=50nxy^{2}+10\left(27n+1\right)xy^{3}+68nxy^{4}+13\left(53n-1\right)x^{2}y^{3}+40nx^{2}y^{4}+774nx^{3}y^{3}+50nx^{3}y^{4},\\ \left(S_{x}S_{y}\right)f\left(x,y\right)=5nxy^{2}+\frac{1}{3}\left(27n+1\right)xy^{3}+nxy^{4}+\frac{1}{6}\left(53n-1\right)x^{2}y^{3}+\frac{1}{4}nx^{2}y^{4}+\frac{1}{9}43nx^{3}y^{3}+\frac{1}{6}nx^{3}y^{4},\\ \left(D_{x}^{\alpha }D_{y}^{\alpha }\right)f\left(x,y\right)=2^{\alpha }10nxy^{2}+3^{\alpha }\left(27n+1\right)xy^{3}+4^{\alpha }4nxy^{4}+6^{\alpha }\left(53n-1\right)x^{2}y^{3}+8^{\alpha }2nx^{2}y^{4}+9^{\alpha }43nx^{3}y^{3}+12^{\alpha }2nx^{3}y^{4},\\ \left(\left(D_{x}D_{y}\right)\left(D_{x}+D_{y}\right)\right)f\left(x,y\right)=60nxy^{2}+12\left(27n+1\right)xy^{3}+80nxy^{4}+30\left(53n-1\right)x^{2}y^{3}+96nx^{2}y^{4}+2322nx^{3}y^{3}+168nx^{3}y^{4},\\ \left(D_{x}S_{y}+S_{x}D_{y}\right)f\left(x,y\right)=25nxy^{2}+\frac{10}{3}\left(27n+1\right)xy^{3}+17nxy^{4}+\frac{13}{6}\left(53n-1\right)x^{2}y^{3}+5nx^{2}y^{4}+86nx^{3}y^{3}+\frac{25}{6}nx^{3}y^{4},\\ \left(S_{x}J\right)f\left(x,y\right)=\frac{20}{3}nx^{2}+\frac{1}{2}\left(27n-1\right)x^{3}+\frac{8}{5}nx^{4}+\frac{2}{5}\left(53n-1\right)x^{5}+15nx^{6}+\frac{4}{7}nx^{7},\\ \;\left(S_{x}JD_{x}D_{y}\right)f\left(x,y\right)=\frac{20}{3}nx^{2}+\frac{3}{4}\left(27n-1\right)x^{3}+\frac{16}{5}nx^{4}+\frac{6}{5}\left(53n-1\right)x^{5}+\frac{403}{6}nx^{6}+\frac{24}{7}nx^{7}. \end{array}$$

From Figure 1, we partitioned the edge for the neighborhood degree-based indices as shown in Table 3.

#### 5.1.3. NM-Polynomial for the Graph of Xanthan Gum

Let *R*_1_ be a molecular graph for xanthan gum; by applying Table 3 in equation (2), we get

(6) $$\begin{array}{c} 10nx^{2}y^{4}+nx^{5}y^{5}+\left(5n+1\right)x^{3}y^{6}+\left(18n+3\right)x^{3}y^{7}+nx^{4}y^{5}+3nx^{4}y^{6}+10nx4y7+nx5y6+\left(2n+1\right)x6y6+\left(26n-1\right)x6y7+\left(18n-1\right)x6y8+\left(23n-1\right)x7y7+\left(19n-2\right)x7y8+4nx8y8. \end{array}$$

#### 5.1.4. Neighborhood Degree-Based TIs of Xanthan Gum Graph Utilizing NM-Polynomial

By using equation (6), we calculated the neighborhood degree-based topological indices for the xanthan gum graph, and the results are as follows:

(7) $$\begin{array}{c} \left(D_{x}+D_{y}\right)f\left(x,y\right)=60nx^{2}y^{4}+8nx^{3}y^{5}+9\left(5n+1\right)x^{3}y^{6}+10\left(18n+3\right)x^{3}y^{7}+9nx^{4}y^{5}+30nx^{4}y^{6}+110nx^{4}y^{7}+11nx^{5}y^{6}+12\left(2n+1\right)x^{6}y^{6}+13\left(26n-1\right)x^{6}y^{7}+14\left(18n-1\right)x^{6}y^{8}+14\left(23n-1\right)x^{7}y^{7}+15\left(19n-2\right)x^{7}y^{8}+64nx^{8}y^{8},\\ \left(D_{x}D_{y}\right)f\left(x,y\right)=80nx^{2}y^{4}+15nx^{3}y^{5}+18\left(5n+1\right)x^{3}y^{6}+21\left(18n+3\right)x^{3}y^{7}+20nx^{4}y^{5}+72nx^{4}y^{6}+280nx^{4}y^{7}+30nx^{5}y^{6}+36\left(2n+1\right)x^{6}y^{6}+42\left(26n-1\right)x^{6}y^{7}+48\left(18n-1\right)x^{6}y^{8}+49\left(23n-1\right)x^{7}y^{7}+56\left(19n-2\right)x^{7}y^{8}+256nx^{8}y^{8},\\ \left({D_{x}}^{2}+{D_{y}}^{2}\right)f\left(x,y\right)=200nx^{2}y^{4}+34nx^{3}y^{5}+45\left(5n+1\right)x^{3}y^{6}+58\left(18n+3\right)x^{3}y^{7}+41nx^{4}y^{5}+156nx^{4}y^{6}+630nx^{4}y^{7}+61nx^{5}y^{6}+72\left(2n+1\right)x^{6}y^{6}+85\left(26n-1\right)x^{6}y^{7}+100\left(18n-1\right)x^{6}y^{8}+98\left(23n-1\right)x^{7}y^{7}+113\left(19n-2\right)x^{7}y^{8}+512nx^{8}y^{8},\\ \left(S_{x}S_{y}\right)f\left(x,y\right)=\frac{5}{4}nx^{2}y^{4}+\frac{1}{15}nx^{3}y^{5}+\frac{1}{18}\left(5n+1\right)x^{3}y^{6}+\frac{1}{21}\left(18n+3\right)x^{3}y^{7}+\frac{1}{20}nx^{4}y^{5}+\frac{1}{8}nx^{4}y^{6}+\frac{5}{14}nx^{4}y^{7}+\frac{1}{30}nx^{5}y^{6}+\frac{1}{36}\left(2n+1\right)x^{6}y^{6}+\frac{1}{42}\left(26n-1\right)x^{6}y^{7}+\frac{1}{48}\left(18n-1\right)x^{6}y^{8}+\frac{1}{49}\left(23n-1\right)x^{7}y^{7}+\frac{1}{56}\left(19n-2\right)x^{7}y^{8}+\frac{1}{16}nx^{8}y^{8},\\ \left(D_{x}^{\alpha }D_{y}^{\alpha }\right)f\left(x,y\right)=8^{\alpha }10nx^{2}y^{4}+15^{\alpha }nx^{5}y^{5}+18^{\alpha }\left(5n+1\right)x^{3}y^{6}+21^{\alpha }\left(18n+3\right)x^{3}y^{7}+20^{\alpha }nx^{4}y^{5}+24^{\alpha }3nx^{4}y^{6}+28^{\alpha }10nx^{4}y^{7}+30^{\alpha }nx^{5}y^{6}+36^{\alpha }\left(2n+1\right)x^{6}y^{6}+42^{\alpha }\left(26n-1\right)x^{6}y^{7}+48^{\alpha }\left(18n-1\right)x^{6}y^{8}+49^{\alpha }\left(23n-1\right)x^{7}y^{7}+56^{\alpha }\left(19n-2\right)x^{7}y^{8}+64^{\alpha }4nx^{8}y^{8},\\ \left(\left(D_{x}D_{y}\right)\left(D_{x}+D_{y}\right)\right)f\left(x,y\right)=480nx^{2}y^{4}+120nx^{3}y^{5}+162\left(5n+1\right)x^{3}y^{6}+210\left(18n+3\right)x^{3}y^{7}+180nx^{4}y^{5}+720nx^{4}y^{6}+3080nx^{4}y^{7}+330nx^{5}y^{6}+432\left(2n+1\right)x^{6}y^{6}+546\left(26n-1\right)x^{6}y^{7}+672\left(18n-1\right)x^{6}y^{8}+686\left(23n-1\right)x^{7}y^{7}+840\left(19n-2\right)x^{7}y^{8}+4096nx^{8}y^{8},\\ \left(D_{x}S_{y}+S_{x}D_{y}\right)f\left(x,y\right)=25nx^{2}y^{4}+\frac{34}{15}nx^{3}y^{5}+\frac{5}{2}\left(5n+1\right)x^{3}y^{6}+\frac{58}{21}\left(18n+3\right)x^{3}y^{7}+\frac{41}{20}nx^{4}y^{5}+\frac{13}{2}nx^{4}y^{6}+\frac{325}{14}nx^{4}y^{7}+\frac{61}{30}nx^{5}y^{6}+2\left(2n+1\right)x^{6}y^{6}+\frac{85}{42}\left(26n-1\right)x^{6}y^{7}+\frac{25}{12}\left(18n-1\right)x^{6}y^{8}+2\left(23n-1\right)x^{7}y^{7}+\frac{113}{56}\left(19n-2\right)x^{7}y^{8}+8nx^{8}y^{8},\\ \left(S_{x}J\right)f\left(x,y\right)=\frac{10}{3}nx^{6}+\frac{1}{4}nx^{8}+\frac{2}{9}\left(6n+1\right)x^{9}+\frac{3}{5}\left(7n+1\right)x^{10}+2nx^{11}+\frac{1}{6}\left(2n+1\right)x^{12}+\frac{2}{13}\left(26n-1\right)x^{13}+\frac{1}{7}\left(41n-2\right)x^{14}+\frac{2}{15}\left(19n-2\right)x^{15}+\frac{1}{2}nx^{16},\\ \;\left(S_{x}JD_{x}D_{y}\right)f\left(x,y\right)=\frac{40}{3}nx^{6}+\frac{15}{8}nx^{8}+\frac{2}{9}\left(55n+9\right)x^{9}+\frac{1}{10}\left(450n+63\right)x^{10}+\frac{310}{11}nx^{11}+3\left(2n+1\right)x^{12}+\frac{42}{13}\left(26n-1\right)x^{13}+\frac{1}{14}\left(1991n-97\right)x^{14}+\frac{56}{15}\left(19n-2\right)x^{15}+16nx^{16}. \end{array}$$

With reference to the molecular structure of xanthan gum shown in Figure 1, the edge partition is obtained. With respect to the edge partition, the M-polynomial and NM-polynomial equations (4) and (6) are generated and applied to get the degree-based and neighborhood degree-based topological index results which was shown in 5.3.2 and 5.3.3. We assign the values for *n* = 1 to 10, resulting in Tables 4 and 5, respectively.

For equations (4) and (6), we show the 3D plots for degree-based and neighborhood degree-based polynomials.

Figure 2(a) represents the neighborhood degree-based topological indices for neighborhood M-polynomial.  Figure 2(b) represents the degree-based topological indices for M-polynomial for xanthan gum.

We now present the degree-based and neighborhood degree-based TIs for gellan gum and polyacrylamide using NM-polynomial and M-polynomial in the same way which was used for xanthan gum graph. The results are as follows:

### 5.2. Gellan Gum

The bacterium Sphingomonas elodea produces the high molecular weight polymer gellan gum, which belongs to the polysaccharide group (see [39, 40]). It is also made up of four molecules: (1,4)-*β*-D-glucuronic acid, (1,3)-*β*-D-glucose, (1,4)-*α*-L-rhamnose, and (1,4)-*β*-D-glucose (see [41]). Delatte [42] discovered the pore-filling ability of gellan gum to reduce permeability and increase strength of shallow soils. Now, we see the structure of gellan gum, which is given Figure 3.

From Figure 3, we partitioned the edge for the degree-based and neighborhood degree-based indices as shown in Tables 6 and 7.

#### 5.2.1. M-Polynomial and NM-Polynomial of Gellan Gum

Let *R*_2_ be a molecular graph for gellan gum; by applying the edge partitions of degree-based and neighborhood degree-based indices in equations (1) and (2), respectively, we get the following results.

(8) $$\begin{array}{c} M\left(R_{2},x,y\right)=2nxy^{2}+\left(11n+2\right)xy^{3}+\left(18n-2\right)x^{2}y^{3}+17nx^{3}y^{3}, \end{array}$$

(9) $$\begin{array}{c} NM\left(R_{2},x,y\right)=2nx^{2}y^{4}+2nx^{3}y^{5}+\left(n+1\right)x^{3}y^{6}+\left(8n+1\right)x^{3}y^{7}+2nx^{4}y^{7}+nx^{5}y^{8}+\left(n+1\right)x^{6}y^{6}+\left(10n-1\right)x^{6}y^{7}+\left(6n-1\right)x^{6}y^{8}+\left(8n+1\right)x^{7}y^{7}+\left(6n-2\right)x^{7}y^{8}+nx^{8}y^{8}. \end{array}$$

#### 5.2.2. Degree-Based TIs of Gellan Gum Graph Utilizing M-Polynomial

By using equation (8), we calculate the degree-based topological indices for the gellan gum graph, and the results are as follows:

- *M*_1_(*G*) = 6*nxy*^2^ + 4(11*n* + 2)*xy*^3^ + 5(18*n* − 2)*x*^2^*y*^3^ + 102*nx*^3^*y*^3^
- *M*_2_(*G*) = 4*nxy*^2^ + 3(11*n* + 2)*xy*^3^ + 6(18*n* − 2)*x*^2^*y*^3^ + 153*nx*^3^*y*^3^
- *F*(*G*) = 10*nxy*^2^ + 10(11*n* + 2)*xy*^3^ + 13(18*n* − 2)*x*^2^*y*^3^ + 306*nx*^3^*y*^3^
-  ^*nm*^*M*_2_(*G*) = *nxy*^2^ + (1/3)(11*n* + 2)*xy*^3^ + (1/3)(18*n* − 2)*x*^2^*y*^3^ + (17/9)*nx*^3^*y*^3^
- *R*_*α*_(*G*) = 2^*α*^2*nxy*^2^ + 3^*α*^(11*n* + 2)*xy*^3^ + 6^*α*^(18*n* − 2)*x*^2^*y*^3^ + 9^*α*^17*nx*^3^*y*^3^
- *ReZG*_3_(*G*) = 12*nxy*^2^ + 12(11*n* + 2)*xy*^3^ + 30(18*n* − 2)*x*^2^*y*^3^ + 918*nx*^3^*y*^3^
- *SDD*(*G*) = 5*nxy*^2^ + (10/3)(11*n* + 2)*xy*^3^ + (13/6)(18*n* − 2)*x*^2^*y*^3^ + 34*nx*^3^*y*^3^
- *H*(*G*) = (4/3)*nx*^3^ + (1/2)(11*n* + 2)*x*^4^ + (2/5)(18*n* − 2)*x*^5^ + (17/3)*nx*^6^
- *I*(*G*) = (4/3)*nx*^3^ + (3/4)(11*n* + 2)*x*^4^ + (6/5)(18*n* − 2)*x*^5^ + (51/2)*nx*^6^

#### 5.2.3. Neighborhood Degree-Based TIs of Gellan Gum Graph Utilizing NM-Polynomial

By using equation (9), we calculate the neighborhood degree-based topological indices for the gellan gum graph, and the results are as follows:

- *NM*_1_(*G*) = 12*nx*^2^*y*^4^ + 16*nx*^3^*y*^5^ + 9(*n* + 1)*x*^3^*y*^6^ + 10(8*n* + 1)*x*^3^*y*^7^ + 22*nx*^4^*y*^7^ + 13*nx*^5^*y*^8^ + 12(*n* + 1)*x*^6^*y*^6^ + 13(10*n* − 1)*x*^6^*y*^7^ + 14(6*n* − 1)*x*^6^*y*^8^ + 14(8*n* + 1)*x*^7^*y*^7^ + 15(6*n* − 2)*x*^7^*y*^8^ + 16*nx*^8^*y*^8^
- *NM*_2_(*G*) = 16*nx*^2^*y*^4^ + 30*nx*^3^*y*^5^ + 18(*n* + 1)*x*^3^*y*^6^ + 21(8*n* + 1)*x*^3^*y*^7^ + 56*nx*^4^*y*^7^ + 40*nx*^5^*y*^8^ + 36(*n* + 1)*x*^6^*y*^6^ + 42(10*n* − 1)*x*^6^*y*^7^ + 48(6*n* − 1)*x*^6^*y*^8^ + 49(8*n* + 1)*x*^7^*y*^7^ + 56(6*n* − 2)*x*^7^*y*^8^ + 64*nx*^8^*y*^8^
- *NF*(*G*) = 40*nx*^2^*y*^4^ + 68*nx*^3^*y*^5^ + 45(*n* + 1)*x*^3^*y*^6^ + 58(8*n* + 1)*x*^3^*y*^7^ + 130*nx*^4^*y*^7^ + 89*nx*^5^*y*^8^ + 72(*n* + 1)*x*^6^*y*^6^ + 85(10*n* − 1)*x*^6^*y*^7^ + 100(6*n* − 1)*x*^6^*y*^8^ + 98(8*n* + 1)*x*^7^*y*^7^ + 113(6*n* − 2)*x*^7^*y*^8^ + 128*nx*^8^*y*^8^
-  ^*nm*^*NM*_2_(*G*) = (1/4)*nx*^2^*y*^4^ + (2/15)*nx*^3^*y*^5^ + (1/18)(*n* + 1)*x*^3^*y*^6^ + (1/21)(8*n* + 1)*x*^3^*y*^7^ + (1/14)*nx*^4^*y*^7^ + (1/40)*nx*^5^*y*^8^ + (1/36)(*n* + 1)*x*^6^*y*^6^ + (1/42)(10*n* − 1)*x*^6^*y*^7^ + (1/48)(6*n* − 1)*x*^6^*y*^8^ + (1/49)(8*n* + 1)*x*^7^*y*^7^ + (1/56)(6*n* − 2)*x*^7^*y*^8^ + (1/64)*nx*^8^*y*^8^
- *NR*_*α*_(*G*) = 8^*α*^2*nx*^2^*y*^4^ + 15^*α*^2*nx*^3^*y*^5^ + 18^*α*^(*n* + 1)*x*^3^*y*^6^ + 21^*α*^(8*n* + 1)*x*^3^*y*^7^ + 28^*α*^2*nx*^4^*y*^7^ + 40^*α*^*nx*^5^*y*^8^ + 36^*α*^(*n* + 1)*x*^6^*y*^6^ + 42^*α*^(10*n* − 1)*x*^6^*y*^7^ + 48^*α*^(6*n* − 1)*x*^6^*y*^8^ + 49^*α*^(8*n* + 1)*x*^7^*y*^7^ + 56^*α*^(6*n* − 2)*x*^7^*y*^8^ + 64^*α*^*nx*^8^*y*^8^
- *ND*_3_(*G*) = 96*nx*^2^*y*^4^ + 240*nx*^3^*y*^5^ + 162(*n* + 1)*x*^3^*y*^6^ + 210(8*n* + 1)*x*^3^*y*^7^ + 616*nx*^4^*y*^7^ + 520*nx*^5^*y*^8^ + 432(*n* + 1)*x*^6^*y*^6^ + 546(10*n* − 1)*x*^6^*y*^7^ + 672(6*n* − 1)*x*^6^*y*^8^ + 686(8*n* + 1)*x*^7^*y*^7^ + 840(6*n* − 2)*x*^7^*y*^8^ + 1024*nx*^8^*y*^8^
- *ND*_5_(*G*) = 5*nx*^2^*y*^4^ + (68/15)*nx*^3^*y*^5^ + (5/2)(*n* + 1)*x*^3^*y*^6^ + (58/7)(8*n* + 1)*x*^3^*y*^7^ + (65/14)*nx*^4^*y*^7^ + (89/40)*nx*^5^*y*^8^ + 2(*n* + 1)*x*^6^*y*^6^ + (85/42)(10*n* − 1)*x*^6^*y*^7^ + (25/12)(6*n* − 1)*x*^6^*y*^8^ + 2(8*n* + 1)*x*^7^*y*^7^ + (113/56)(6*n* − 2)*x*^7^*y*^8^ + 2*nx*^8^*y*^8^
- *NH*(*G*) = (2/3)*nx*^6^ + (1/2)*nx*^8^ + (2/9)(*n* + 1)*x*^9^ + (2/10)(8*n* + 1)*x*^10^ + (4/11)*nx*^11^ + (1/6)(*n* + 1)*x*^12^ + (2/13)(11*n* − 1)*x*^13^ + 2*nx*^14^ + (2/15)(6*n* − 2)*x*^15^ + (1/8)*nx*^16^
- *NI*(*G*) = (8/3)*nx*^6^ + (15/4)*nx*^8^ + 2(*n* + 1)*x*^9^ + (21/10)(8*n* + 1)*x*^10^ + (56/11)*nx*^11^ + 3(*n* + 1)*x*^12^ + (2/13)(230*n* − 21)*x*^13^ + (1/14)(680*n* + 1)*x*^14^ + (56/15)(6*n* − 2)*x*^15^ + 4*nx*^16^

With reference to the molecular structure of gellan gum shown in Figure 3, the edge partition is obtained. With respect to the edge partition, the M-polynomial and NM-polynomial equations (??) and (9) are generated and applied to get the degree-based and neighborhood degree-based topological index results which was shown in 5.3.2 and 5.3.3. We assign the values for *n* = 1 to 10, resulting in Tables 8 and 9, respectively.

For equations (8) and (9), we show the 3D plots for degree-based and neighborhood degree-based polynomials.

Figure 4(a) represents the neighborhood degree-based topological indices for neighborhood M-polynomial.  Figure 4(b) represents the degree-based topological indices for M-polynomial for gellan gum.

### 5.3. Polyacrylamide

A water-soluble polymer is called polyacrylamide (PAM).  Figure 5 demonstrates the PAM structural unit. Considering that it is more efficient and reasonably priced, it is frequently utilized for EOR, water treatment, and soil amendment effects (see [43–45]). The dynamic property discovered by Im et al. [46] is increased flocculation effectiveness and total durability of PAM solution for agricultural purposes to help reduce water corrosion. Now, we see the structure of polyacrylamide, which is given in Figure 5.

From Figure 5, we partitioned the edge for the degree-based and neighborhood degree-based indices, respectively, which are given in Tables 10 and 11.

#### 5.3.1. M-Polynomial and NM-Polynomial of Polyacrylamide

Let *R*_3_ be a molecular graph for polyacrylamide; by applying the edge partitions of degree-based and neighborhood degree-based indices in equations (1) and (2), respectively, we get the following results.

(10) $$\begin{array}{c} M\left(R_{3},x,y\right)=xy^{2}+\left(4n+1\right)xy^{3}+\left(n-1\right)x^{2}y^{2}+\left(4n-1\right)x^{2}y^{3}+2nx^{3}y^{3}, \end{array}$$

(11) $$\begin{array}{c} NM\left(R_{3},x,y\right)=x^{2}y^{4}+4nx^{3}y^{5}+x^{3}y^{6}+x^{4}y^{7}+\left(n-1\right)x^{5}y^{5}+x^{5}y^{6}+\left(4n-3\right)x^{5}y^{7}+x^{6}y^{6}+\left(2n+1\right)x^{6}y^{7}. \end{array}$$

#### 5.3.2. Degree-Based TIs of Polyacrylamide Graph Utilizing M-Polynomial

By using equation (10), we calculate the degree-based topological indices for the molecular graph of polyacrylamide, and the results are as follows:

- *M*_1_(*G*) = 3*xy*^2^ + 4(4*n* + 1)*xy*^3^ + 4(*n* − 1)*x*^2^*y*^2^ + 5(4*n* − 1)*x*^2^*y*^3^ + 12*nx*^3^*y*^3^
- *M*_2_(*G*) = 2*xy*^2^ + 3(4*n* + 1)*xy*^3^ + 4(*n* − 1)*x*^2^*y*^2^ + 6(4*n* − 1)*x*^2^*y*^3^ + 18*nx*^3^*y*^3^
- *F*(*G*) = 5*xy*^2^ + 10(4*n* + 1)*xy*^3^ + 8(*n* − 1)*x*^2^*y*^2^ + 13(4*n* − 1)*x*^2^*y*^3^ + 36*nx*^3^*y*^3^
-  ^*nm*^*M*_2_(*G*) = (1/2)*xy*^2^ + (1/3)(4*n* + 1)*xy*^3^ + (1/4)(*n* − 1)*x*^2^*y*^2^ + (1/6)(4*n* − 1)*x*^2^*y*^3^ + (2/9)*nx*^3^*y*^3^
- *R*_*α*_(*G*) = 2^*α*^*xy*^2^ + 3^*α*^(4*n* + 1)*xy*^3^ + 4^*α*^(*n* − 1)*x*^2^*y*^2^ + 6^*α*^(4*n* − 1)*x*^2^*y*^3^ + 9^*α*^2*nx*^3^*y*^3^
- *ReZG*_3_(*G*) = 6*xy*^2^ + 12(4*n* + 1)*xy*^3^ + 16(*n* − 1)*x*^2^*y*^2^ + 30(4*n* − 1)*x*^2^*y*^3^ + 108*nx*^3^*y*^3^
- *SDD*(*G*) = (5/2)*xy*^2^ + (10/3)(4*n* + 1)*xy*^3^ + 2(*n* − 1)*x*^2^*y*^2^ + (13/6)(4*n* − 1)*x*^2^*y*^3^ + 4*nx*^3^*y*^3^
- *H*(*G*) = (2/3)*x*^3^ + (1/2)(4*n* + 1)*x*^4^ + (1/2)(*n* − 1)*x*^4^ + (2/5)(4*n* − 1)*x*^5^ + (2/3)*nx*^6^
- *I*(*G*) = (2/3)*x*^3^ + (3/4)(4*n* + 1)*x*^4^ + (*n* − 1)*x*^4^ + (6/5)(4*n* − 1)*x*^5^ + 3*nx*^6^

#### 5.3.3. Neighborhood Degree-Based TIs of Polyacrylamide Graph Utilizing NM-Polynomial

By using equation (11), we calculate the neighborhood degree-based topological indices for the molecular graph of polyacrylamide, and the results are as follows:

- *NM*_1_(*G*) = 6*x*^2^*y*^4^ + 32*nx*^3^*y*^5^ + 9*x*^3^*y*^6^ + 11*x*^4^*y*^7^ + 10(*n* − 1)*x*^5^*y*^5^ + 11*x*^5^*y*^6^ + 12(4*n* − 3)*x*^5^*y*^7^ + 12*x*^6^*y*^6^ + 13(2*n* + 1)*x*^6^*y*^7^
- *NM*_2_(*G*) = 8*x*^2^*y*^4^ + 60*nx*^3^*y*^5^ + 18*x*^3^*y*^6^ + 28*x*^4^*y*^7^ + 25(*n* − 1)*x*^5^*y*^5^ + 30*x*^5^*y*^6^ + 35(4*n* − 3)*x*^5^*y*^7^ + 36*x*^6^*y*^6^ + 42(2*n* + 1)*x*^6^*y*^7^
- *NF*(*G*) = 20*x*^2^*y*^4^ + 136*nx*^3^*y*^5^ + 45*x*^3^*y*^6^ + 65*x*^4^*y*^7^ + 50(*n* − 1)*x*^5^*y*^5^ + 61*x*^5^*y*^6^ + 74(4*n* − 3)*x*^5^*y*^7^ + 72*x*^6^*y*^6^ + 85(2*n* + 1)*x*^6^*y*^7^
-  ^*nm*^*NM*_2_(*G*) = (1/8)*x*^2^*y*^4^ + (4/15)*nx*^3^*y*^5^ + (1/18)*x*^3^*y*^6^ + (1/28)*x*^4^*y*^7^ + (1/25)(*n* − 1)*x*^5^*y*^5^ + (1/30)*x*^5^*y*^6^ + (1/35)(4*n* − 3)*x*^5^*y*^7^ + (1/36)*x*^6^*y*^6^ + (1/42)(2*n* + 1)*x*^6^*y*^7^
- *NR*_*α*_(*G*) = 8^*α*^*x*^2^*y*^4^ + 15^*α*^4*nx*^3^*y*^5^ + 18^*α*^*x*^3^*y*^6^ + 28^*α*^*x*^4^*y*^7^ + 25^*α*^(*n* − 1)*x*^5^*y*^5^ + 30^*α*^*x*^5^*y*^6^ + 35^*α*^(4*n* − 3)*x*^5^*y*^7^ + 36^*α*^*x*^6^*y*^6^ + 42^*α*^(2*n* + 1)*x*^6^*y*^7^
- *ND*_3_(*G*) = 48*x*^2^*y*^4^ + 480*nx*^3^*y*^5^ + 162*x*^3^*y*^6^ + 308*x*^4^*y*^7^ + 250(*n* − 1)*x*^5^*y*^5^ + 330*x*^5^*y*^6^ + 420(4*n* − 3)*x*^5^*y*^7^ + 432*x*^6^*y*^6^ + 546(2*n* + 1)*x*^6^*y*^7^
- *ND*_5_(*G*) = (5/2)*x*^2^*y*^4^ + (136/15)*nx*^3^*y*^5^ + (5/2)*x*^3^*y*^6^ + (65/28)*x*^4^*y*^7^ + 2(*n* − 1)*x*^5^*y*^5^ + (61/30)*x*^5^*y*^6^ + (74/35)(4*n* − 3)*x*^5^*y*^7^ + 2*x*^6^*y*^6^ + (85/42)(2*n* + 1)*x*^6^*y*^7^
- *NH*(*G*) = (1/3)*x*^6^ + *nx*^8^ + (2/9)*x*^9^ + (1/5)(*n* − 1)*x*^10^ + (4/11)*x*^11^ + (1/3)(2*n* − 1)*x*^12^ + (2/13)(2*n* + 1)*x*^13^
- *NI*(*G*) = (4/3)*x*^6^ + (15/8)*nx*^8^ + 2*x*^9^ + (5/2)(*n* − 1)*x*^10^ + (58/11)*x*^11^ + (1/3)(35*n* − 26)*x*^12^ + (1/13)(2*n* + 1)*x*^13^

With reference to the molecular structure of polyacrylamide shown in Figure 5, the edge partition is obtained. With respect to the edge partition, the M-polynomial and NM-polynomial equations (10) and (11) are generated and applied to get the degree-based and neighborhood degree-based topological index results which was shown in 5.3.2 and 5.3.3. We assign the values for “*n*” in those results as *n* = 1 to 10, resulting in Tables 12 and 13, respectively.

For equations (10) and (11), we show the 3D plots for degree-based and neighborhood degree-based polynomials.

Figure 6(a) represents the neighborhood degree-based topological indices for neighborhood M-polynomial, and Figure 6(b) represents the degree-based topological indices for M-polynomial for polyacrylamide.

The surface view of Figures 2, 4, and 6 represents the 3D plots of NM-polynomial and M-polynomial of xanthan gum, gellan gum, and polyacrylamide, respectively. We show the 3D plots with the range of *x* and *y* axes taken arbitrarily from -10 to 10; except for the vertical axis values, no change would appear in the figures for the higher and lower ranges. It shows the changes of the M-polynomial and NM-polynomial for varying its arguments.

The graphical representation of Figures 7(a), 7(c), and 7(e) represents the M-polynomial of degree-based topological indices for xanthan gum, gellan gum, and polyacrylamide which is derived from Tables 4, 8, and 12, respectively. Similarly, Figures 7(b), 7(d), and 7(f) represent the NM-polynomial of neighborhood degree-based topological indices for xanthan gum, gellan gum, and polyacrylamide which is derived from Tables 5, 9, and 13, respectively.

## 6. Conclusion

In this paper, we examine the structures of three biopolymers: xanthan gum, gellan gum, and polyacrylamide. First, we obtained the M-polynomial and NM-polynomial of the molecular graphs of those biopolymers. Later, for the structures under consideration, some degree-based and neighborhood degree-based indices, such as the first Zagreb index, the second Zagreb index, the modified second Zagreb index, the third redefined Zagreb index, the forgotten index, the Randic index, the inverse Randic index, the symmetric division index, the inverse sum index, the harmonic index, and their neighborhood versions, were derived using M-polynomial and NM-polynomial, respectively. A graphic interpretation and comparison of the findings are done. Understanding the topology of the aforementioned biopolymer structures is made easier by this work. In future work, we will consider comparing the physicochemical characteristics of distinct chemical compounds to the forecasting power of neighborhood degree-based topological indices.

## Figures and Tables

**Figure 1:** Representation of the structure of xanthan gum.

**Figure 2:** 3D plots of NM-polynomial and M-polynomial of xanthan gum.

**Figure 3:** The structure of gellan gum.

**Figure 4:** 3D plots of NM-polynomial and M-polynomial of gellan gum.

**Figure 5:** The structure of polyacrylamide.

**Figure 6:** 3D plots of NM-polynomial and M-polynomial of polyacrylamide.

**Figure 7:** Graphical representation for several M-polynomial and NM-polynomials utilizing TIs for xanthan gum, gellan gum, and polyacrylamide.

**Table 1:** The correlation between several TIs with M-polynomial and NM-polynomial.

TI	Formula *g*(*δ*_*u*_, *δ*_*v*_)	Derivative from *h*(*x*, *y*) = *M*(*R*; *x*, *y*) or *NM*(*R*; *x*, *y*)
*M*_1_/*NM*_1_	$\underset{vu\in E\left(G\right)}{\sum }\left(\delta_{u}+\delta_{v}\right)$	(*D*_*x*_ + *D*_*y*_)(*h*(*x*, *y*))_*x*=*y*=1_
*M*_2_/*NM*_2_	$\underset{vu\in E\left(G\right)}{\sum }\left(\delta_{u}\times \delta_{v}\right)$	(*D*_*x*_*D*_*y*_)(*h*(*x*, *y*))_*x*=*y*=1_
*F*/*NF*	$\underset{vu\in E\left(G\right)}{\sum }\left({\delta_{u}}^{2}+{\delta_{v}}^{2}\right)$	(*D*_*x*_^2^ + *D*_*y*_^2^)(*h*(*x*, *y*))_*x*=*y*=1_
_ _^*m*^ *M*_2_/^*nm*^*M*_2_	$\underset{vu\in E\left(G\right)}{\sum }\frac{1}{\left(\delta_{u}.\delta_{v}\right)}$	(*S*_*x*_*S*_*y*_)(*h*(*x*, *y*))_*x*=*y*=1_
*R*_*α*_/*NR*_*α*_	$\underset{vu\in E\left(G\right)}{\sum }{\left[\delta_{u}\delta_{v}\right]}^{\alpha }$	(*D*_*x*_^*α*^*D*_*y*_^*α*^)(*h*(*x*, *y*))_*x*=*y*=1_
*ReZG*_3_/*ND*_3_	$\underset{vu\in E\left(G\right)}{\sum }\left(\delta_{u}+\delta_{v}\right)\left(\delta_{u}.\delta_{v}\right)$	((*D*_*x*_*D*_*y*_)(*D*_*x*_ + *D*_*y*_))(*h*(*x*, *y*))_*x*=*y*=1_
*SDD*/*ND*_5_	$\underset{vu\in E\left(G\right)}{\sum }\left(\frac{\delta_{u}^{2}+\delta_{v}^{2}}{\delta_{u}.d\delta_{v}}\right)$	(*D*_*x*_*S*_*y*_ + *S*_*x*_*D*_*y*_)(*h*(*x*, *y*))_*x*=*y*=1_
*H*/*NH*	$\underset{vu\in E\left(G\right)}{\sum }\frac{2}{\delta_{u}+\delta_{v}}$	(*S*_*x*_*J*)(*h*(*x*, *y*))_*x*=*y*=1_
*I*/*NI*	$\underset{vu\in E\left(G\right)}{\sum }\frac{\delta_{u}.\delta_{v}}{\delta_{u}+\delta_{v}}$	(*S*_*x*_*JD*_*x*_*D*_*y*_)(*h*(*x*, *y*))_*x*=*y*=1_

**Table 2:** Edge partition of the degree-based indices for xanthan gum graph.

(*d*_*u*_, *d*_*v*_), *uv* ∈ *E*(*G*)	No. of edges
(1,2)	10*n*
(1,3)	27*n* + 1
(1,4)	4*n*
(2,3)	53*n* − 1
(2,4)	2*n*
(3,3)	43*n*
(3,4)	2*n*

**Table 3:** Edge partition of the neighborhood degree-based indices for xanthan gum graph.

(*nd*_*u*_, *nd*_*v*_), *uv* ∈ *E*(*G*)	No. of edges
(2,4)	10*n*
(3,5)	*n*
(3,6)	5*n* + 1
(3,7)	18*n* + 3
(4,5)	*n*
(4,6)	3*n*
(4,7)	10*n*
(5,6)	*n*
(6,6)	2*n* + 1
(6,7)	26*n* − 1
(6,8)	18*n* − 1
(7,7)	23*n* − 1
(7,8)	19*n* − 2
(8,8)	4*n*

**Table 4:** Xanthan gum's degree-based indices for the notation of *n* = 1 to 10.

[*n*]	*M*_1_	*M*_2_	*F*	^*m*^*M*_2_	*R*	*ReZG*_3_	*SDD*	*H*	*I*
1	706	859	1938	29.19	62.08	4622	343.17	58.64	163.86
2	1413	1721	3879	58.22	124.00	9262	685.17	117.18	328.17
3	2120	2583	5820	87.25	185.91	13902	1027.17	175.71	492.49
4	2827	3445	7761	116.28	247.83	18542	1369.17	234.25	656.80
5	3534	4307	9702	145.31	309.74	23182	1711.17	292.79	821.11
6	4241	5169	11643	174.33	371.66	27822	2053.17	351.33	985.42
7	4948	6031	13584	203.36	433.57	32462	2395.17	409.87	1149.73
8	5655	6893	15525	232.39	495.48	37102	2737.17	468.40	1314.05
9	6362	7755	17466	261.42	557.40	41742	3079.17	526.94	1478.36
10	7069	8617	19407	290.44	619.31	46382	3421.17	585.48	1642.67

**Table 5:** Xanthan gum's neighborhood degree-based indices for the notation of *n* = 1 to 10.

[*n*]	*NM*_1_	*NM*_2_	*NF*	_ _^*nm*^ *NM*_2_	*NR*	*ND*_3_	*ND*_5_	*NH*	*NI*
1	1718	5306	11240	5.06	25.05	70130	312.38	24.62	413.43
2	3456	10746	22698	10.00	49.75	142620	622.12	48.96	833.19
3	5194	16186	34156	14.94	74.45	215110	931.85	73.30	1252.95
4	6932	21626	45614	19.88	99.15	287600	1241.59	97.64	1672.71
5	8670	27066	57072	24.81	123.86	360090	1551.33	121.99	2092.47
6	10408	32506	68530	29.75	148.56	432580	1861.06	146.33	2512.23
7	12146	37946	79988	34.69	173.26	505070	2170.80	170.67	2931.99
8	13884	43386	91446	39.63	197.96	577560	2480.54	195.01	3351.75
9	15622	48826	102904	44.57	222.66	650056	2790.28	219.35	3771.51
10	17360	54266	114362	49.50	247.36	722540	3100.01	243.69	4191.27

**Table 6:** Edge partition of the degree-based indices for gellan gum graph.

(*d*_*u*_, *d*_*v*_), *uv* ∈ *E*(*G*)	No. of edges
(1,2)	2*n*
(1,3)	11*n* + 2
(2,3)	18*n* − 2
(3,3)	17*n*

**Table 7:** Edge partition of the neighborhood degree-based indices for gellan gum graph.

(*nd*_*u*_, *nd*_*v*_), *uv* ∈ *E*(*G*)	No. of edges
(2,4)	2*n*
(3,5)	2*n*
(3,6)	*n* + 1
(3,7)	8*n* + 1
(4,7)	2*n*
(5,8)	*n*
(6,6)	*n* + 1
(6,7)	10*n* − 1
(6,8)	6*n* − 1
(7,7)	8*n* + 1
(7,8)	6*n* − 2
(8,8)	*n*

**Table 8:** Gellan gum's degree-based indices for the notation of *n* = 1 to 10.

[*n*]	*M*_1_	*M*_2_	*F*	_ _^*nm*^ *M*_2_	*R*	*ReZG*_3_	*SDD*	*H*	*I*
1	240	292	654	11.22	21.12	1566	117.0	19.9	55.78
2	482	590	1314	22.28	41.90	3168	231.7	39.6	112.47
3	724	888	1974	33.33	62.68	4770	346.3	59.3	169.15
4	966	1186	2634	44.39	83.46	6372	461.0	79.0	225.83
5	1208	1484	3294	55.44	104.24	7974	575.7	98.7	282.52
6	1450	1782	3954	66.50	125.02	9576	690.3	118.4	339.20
7	1692	2080	4614	77.56	145.80	11178	805.0	138.1	395.88
8	1934	2378	5274	88.61	166.58	12780	919.7	157.8	452.57
9	2176	2676	5934	99.67	187.36	14382	1034.3	177.5	509.25
10	2418	2974	6594	110.72	208.14	15984	1149.0	197.2	565.93

**Table 9:** Gellan gum's neighborhood degree-based indices for the notation of *n* = 1 to 10.

[*n*]	*NM*_1_	*NM*_2_	*NF*	_ _^*nm*^ *NM*_2_	*NR*	*ND*_3_	*ND*_5_	*NH*	*NI*
1	584	1786	3810	1.66	10.77	23382	3964.68	8.30	140.14
2	1180	3650	7758	3.26	21.33	48172	15818.71	16.44	283.80
3	1176	5514	11706	4.85	31.90	72962	35568.74	24.58	427.26
4	2372	7378	15654	6.44	42.47	97752	63214.77	32.71	571.13
5	2968	9242	19602	8.04	53.04	122542	98756.80	40.85	714.79
6	3564	11106	23550	9.63	63.61	147332	142194.84	48.99	858.46
7	4160	12970	27498	11.22	74.18	172122	193528.87	57.12	1002.12
8	4756	14834	31446	12.82	84.75	196912	252758.90	65.26	1145.78
9	5352	16698	35394	14.41	95.31	221702	319884.93	73.40	1289.45
10	5948	18562	39342	16.00	105.88	246492	394906.96	81.53	1433.11

**Table 10:** Edge partition of the degree-based indices for polyacrylamide.

(*d*_*u*_, *d*_*v*_), *uv* ∈ *E*(*G*)	No. of edges
(1,2)	1
(1,3)	4*n* + 1
(2,2)	*n* − 1
(2,3)	4*n* − 1
(3,3)	2*n*

**Table 11:** Edge partition of the neighborhood degree-based indices for polyacrylamide.

(*nd*_*u*_, *nd*_*v*_), *uv* ∈ *E*(*G*)	No. of edges
(2,4)	1
(3,5)	4*n*
(3,6)	1
(4,7)	1
(5,5)	*n* − 1
(5,6)	1
(5,7)	4*n* − 3
(6,6)	1
(6,7)	2*n* + 1

**Table 12:** Polyacrylamide's degree-based indices for the notation of *n* = 1 to 10 with the comparison of numbers.

[*n*]	*M*_1_	*M*_2_	*F*	^*nm*^*M*_2_	*R*	*ReZG*_3_	*SDD*	*H*	*I*
1	50	53	130	2.89	5.49	264	29.67	5.03	11.02
2	105	113	271	5.86	10.59	562	60.17	10.47	23.48
3	160	173	412	8.83	15.70	860	90.67	15.90	35.95
4	215	233	553	11.81	20.81	1158	121.17	21.33	48.42
5	270	293	694	14.78	25.92	1456	151.67	26.77	60.88
6	325	353	835	17.75	31.03	1754	182.17	32.20	73.35
7	380	413	976	20.72	36.14	2052	212.67	37.63	85.82
8	435	473	1117	23.69	41.25	2350	243.17	43.07	98.28
9	490	533	1258	26.67	46.36	2648	273.67	48.50	110.75
10	545	593	1399	29.64	51.47	2946	304.17	53.93	123.22

**Table 13:** Polyacrylamide's neighborhood degree-based indices for the notation of *n* = 1 to 10 with the comparison of numbers.

[*n*]	*NM*_1_	*NM*_2_	*NF*	^*nm*^*NM*_2_	*NR*	*ND*_3_	*ND*_5_	*NH*	*NI*
1	132	341	728	0.64	2.79	3818	28.61	2.71	19.34
2	248	650	1380	1.11	5.01	7320	52.18	4.89	41.16
3	364	959	2032	1.58	7.23	10822	75.75	7.06	62.98
4	480	1268	2684	2.05	9.44	14324	99.32	9.24	84.80
5	596	1577	3336	2.52	11.66	17826	122.89	11.41	106.62
6	712	1886	3988	2.99	13.88	21328	146.46	13.59	128.44
7	828	2195	4640	3.46	16.10	24830	170.04	15.76	150.26
8	944	2504	5292	3.92	18.31	28332	193.61	17.93	172.08
9	1060	2813	5944	4.39	20.53	31834	217.18	20.11	193.90
10	1176	3122	6596	4.86	22.75	35336	240.75	22.28	215.72

## Data Availability

The data used to support the findings of this study are cited at relevant places within the article as references.
